# Cognitive Rehabilitation: Mild Traumatic Brain Injury and Relevance of OTPF

**DOI:** 10.1155/2023/8135592

**Published:** 2023-05-29

**Authors:** Asha Vas, Anna Luedtke, Eryn Ortiz, Natalie Mackie, Samantha Gonzalez

**Affiliations:** ^1^School of Occupational Therapy, Texas Woman's University, Dallas, TX 75235, USA; ^2^Baylor Scott & White Medical Center, Dallas, Texas, USA; ^3^Thrive Skilled Pediatric Care, Dallas, Texas, USA

## Abstract

There is increased awareness of the long-term cognitive sequelae of mild traumatic brain injury (mTBI). Therefore, researchers and clinicians have developed and tested cognitive training protocols to address these challenges. The current review summarized literature that examined existing cognitive rehabilitation/training programs. Specifically, the review listed the impact of these programs on functional domains informed by the Occupational Therapy Practice Framework (OTPF). Literature between the years 2008 and 2022 was gathered from nine databases. Results indicate that several cognitive rehabilitation programs have proven to positively influence domains of occupation, client factors, performance, and context. Occupational therapy practitioners have an opportunity to engage in mTBI management. Furthermore, adopting domains of OTPF may guide assessments, treatment planning, and long-term follow-up.

## 1. Introduction

Over a million Americans sustain a mild traumatic brain injury (mTBI) every year [1]. Mild TBI is defined as an injury to the head with loss of consciousness for 30 minutes or less with posttraumatic amnesia as well as alteration of consciousness for no more than 24 hours with no identifiable lesions on the individual's scans [2]. In the last decade, TBI has received more attention as combat and sports-related activities have led to brain injuries and received extensive news coverage. It is likely that there are a high number of individuals who have experienced a brain injury but have not been diagnosed [3]. Unfortunately, mTBI symptoms are commonly unrecognized and can cause chronic impairments such as attention deficits, headaches, fatigue, posttraumatic stress symptoms, and deficits in executive functioning, all of which negatively impact daily functioning [1]. Approximately 70% of TBIs are considered mTBI and are usually diagnosed after complaints by the individual without postinjury objective findings [4, 5]. It is often easy to mistake mTBI symptoms as they present similarly to stressors such as pain, medication, posttraumatic stress, anxiety, and depression [6].

While some may not experience long-term mTBI-related symptoms, a large number of individuals are increasingly reporting cognitive, physical, and psychological symptoms months and years postinjury [1, 7]. One of the chronic symptoms of mTBI is impaired executive functioning causing difficulties in holding attention, remembering information, and organization and planning [8]. In addition to these issues, it is often difficult for an individual with TBI to maintain employment due to their executive functioning deficits, significantly affecting the learning of job tasks, concentration, and overall job performance [9]. Increased awareness of the long-term cognitive sequelae of mTBI has led to the development of several cognitive rehabilitation training protocols. The American Congress of Rehabilitation Medicine defines cognitive rehabilitation as “a systematic, functionally oriented service of therapeutic activities that is based on assessment and understanding of the patient's brain-behavioral deficits” [10].

Cognitive rehabilitation is designed to use compensatory and rehabilitative mechanisms to improve cognitive function [8]. It is important to tailor cognitive rehabilitation in the context of real-life issues, daily tasks, and functional activities for the individual [11]. The aim of this scoping review is to map cognitive training/rehabilitation programs focused on mitigating cognitive impairments in adults with mTBI. The review selected training programs that either used daily life-relevant assessments, treatments, and/or outcomes of a training program. Additionally, the findings of the review were mapped to align with the domains of the Occupational Therapy Practice Framework (OTPF) [12]. The OTPF guides occupational therapy practice in conjunction with the knowledge and evidence relevant to occupation and occupational therapy within the identified areas of practice and with the appropriate clients. Thus, the OTF helps examine the complex relationship between cognition and tasks of daily living. Furthermore, OTPF–4 is often considered a valuable tool in the academic preparation of students, communication with the public and policymakers, and provision of language that can shape and be shaped by research.

## 2. Method

The current scoping review is aimed at presenting an overview of existing cognitive training programs for adults with mTBI. We adopted Arksey and O'Malley's (2005) methodological framework. The present scoping review included four steps: (1) identifying relevant publications; (2) selecting publications on the basis of predefined inclusion criteria; (3) charting data; and (4) collating, summarizing, and reporting results [13, 14]. The PRISMA (Preferred Reporting Items for Systematic Reviews and Meta-Analyses) model in Figure 1 illustrates the articles screened and included in the scoping review. The OTPF was adopted to summarize the results. The reviewers identified two broad keywords: mTBI and functional cognition. A broad definition of mTBI was adopted for this review. Inclusion of mTBI in research studies that were either based on Glasgow Coma Scale scores and/or self-reports and/or level of functional challenges was included in the review. Additional criteria included the chronic stage of rehabilitation, and adult populations, who were at least three months post mTBI. The broad definition of functional cognition included studies that had functionally relevant rehabilitation assessments and/or training approaches. Therefore, the search string terms included “executive functions” OR “functional cognition” OR “cognitive rehabilitation” OR “cognitive remediation” OR “cognitive training”) AND (“acquired brain injury” OR “traumatic brain injury”).

Electronic databases including CINAHL, PubMed, Nursing and Allied Health, Scopus, Trip, PsychInfo, Cochrane, Web of Science, and Ovid Emcare were used for this scoping review. Literature was limited to studies published in English in the last 15 years between 2008 and 2022. Since cognitive training is conducted at varied sites, we included studies that were conducted in both inpatient and outpatient settings. The scoping search was performed during 2016-2023. Abstracts from the searches were compiled, duplicates were eliminated, and two reviewers (first and second authors) independently screened all original abstracts. Any abstract identified as relevant by either author was brought to the full-text stage. The two authors independently reviewed the full texts, and the final study inclusion required agreement by both authors. Any disagreement on study selection was settled by deliberations ending in consensus. A third reviewer resolved any disagreements among the two reviewers regarding study inclusion/exclusion. A hand search was conducted for any published articles that met the criteria but did not appear in the database. Journals from 2008 to 2022 were searched including the American Journal of Occupational Therapy, Australian Journal of Occupational Therapy, British Journal of Occupational Therapy, and Journal of Head Trauma Rehabilitation.

## 3. Results

The search yielded 8,650 citations (Figure 1); 188 from CINAHL, 250 from PubMed, 330 from Nursing and Allied Health, 2,809 from Scopus, 990 from Trip, 1,215 from PsychInfo, 312 from Cochrane, 1,894 from Web of Science, and 662 from Ovid Emcare (Figure 1, Table 1). The review found several cognitive rehabilitation/training for mTBI populations (Table 2). The findings present integrative approaches of cognitive rehabilitation strategies including remediation, compensation, and relearning of daily functional tasks. In large part, these studies were conducted by rehabilitation professionals (e.g., occupational therapy practitioners, speech pathologists, and neuropsychologists).

The training programs' content and findings were reviewed in light of the domains proposed by the OTPF. The OTPF describes the central domains that ground occupational therapy practice and builds a common understanding of the basic tenets and vision of the profession. The interrelated domains are occupations, contexts, performance patterns, performance skills, and client factors. The purpose of a framework is to provide a structure or base on which to build a system or a concept [12]. As stated in Table 2, the majority of cognitive rehabilitation/training programs align with the domains of occupation and client factors, followed by performance skills, performance patterns, and context. The alignment of the cognitive rehabilitation/training programs with the OTPF domains is based solely on the authors' (reviewers') interpretation of the research studies.

## 4. Discussion

Mild TBI could result in not-so-mild functional challenges, especially in chronic stages of recovery. It is encouraging to see the number of training programs targeting mTBI-related cognitive challenges. The majority of the studies included in this literature review were conducted by a mix of rehabilitation professionals including occupational therapy practitioners, speech pathologists, cognitive scientists, neuropsychologists, and physiatrists. Findings from the review suggest that cognitive training may facilitate improvements in both trained and untrained domains of functioning. All training programs addressed elements of the functional domains that occupational therapy practitioners' address often use in their daily practice. Therefore, we aligned the findings with the OTPF domains. Several training programs (e.g., SMART and CO-OP, [15, 33]) focused on occupation.

*Occupation* is defined as “the everyday activities that people do as individuals, in families, and in communities to occupy time and bring meaning and purpose to life. Occupations include things people need to, want to, and are expected to do” [36]. Occupations are categorized as activities of daily living, instrumental activities of daily living, health management, rest and sleep, education, work, play, leisure, and social participation. Helping individuals improve educational skills [15, 16] or focusing on IADLs [33] leads to significant gains in executive functioning. Similarly, focusing on performance patterns (e.g., GMT [1]) led to gains in executive functions.

*Performance patterns* include habits, routines, roles, and rituals that may be associated with different lifestyles and used in the process of engaging in occupations or activities that support or hinder occupational performance. An example of this would be using a planner to compensate for executive dysfunction and memory deficits as seen in Cognitive Strategy Training [20].

*Performance skills* are observable, goal-directed actions that result in a client's quality of performing desired occupations. Training programs with a component of performance skills (e.g., metacognitive strategy instruction, [25]) work on motor process and social interaction skills. Social interaction in particular can be difficult following an mTBI. One training program working on social communication is cognitive communication. This program uses functional language in the individual's true environment to relearn social skills such as listening, speaking slowly, and fluency [28].

*Client factors* include (1) values, beliefs, and spirituality; (2) body functions; and (3) body structures. Client factors reside within the client and influence the client's performance in occupations. All the training programs (e.g. CogSMART [9] and CST [20]) had some components utilizing client factors since it encompasses both specific and global mental functions. These cognitive functions are critical for daily life activities.

*Context* is a broad construct that encompasses environmental factors and personal factors. Environmental factors include the surroundings of the person, both physical and social, while personal factors include distinct characteristics and backgrounds of the individual. Context can hinder healing as some individuals can be more resistant to therapy than others. Training programs that work on context (e.g., GOALS [22]) work on applying skills to real-life settings.

An mTBI is a chronic health condition and not an isolated event or incident in terms of treatment considerations [37, 38]. Cognitive sequelae of mTBI can endure and even worsen over time when there is no further cognitive monitoring or intervention. These impairments significantly affect long-term functionality [39–41]. Occupational therapy practitioners are in an advantageous position to use OTPF domains to guide and improve functional cognition, that is, the way “an individual utilizes and integrates his or her thinking and processing skills to accomplish everyday activities in clinical and community living environments” [12]. Using the OTPF to examine cognition and cognitive rehabilitation could be one of several ways to strengthen functional cognition.

### 4.1. Clinical Implications for Occupational Therapy

Occupational therapy practice emphasizes the occupational nature of humans [42]. The OTPF's classification guides practitioners to characterize, examine, and guide clients' participation in daily living, which results from the dynamic intersection of clients, their desired engagements, and their contexts (including environmental and personal factors; [43–45]. Functionally, relevant cognitive rehabilitation can help distinguish occupational therapist (OT) practice from that of other professionals, as occupational therapy practitioners use occupation as a medium of treatment and an agent of change. Examining the impact of mTBI on the domains of OTPF could assist in the screening process in primary care or acute-stage rehabilitation settings. In addition to standardized cognitive assessments, OTPF domain/domain-specific assessments could assist in establishing a comprehensive baseline prior to starting occupational therapy.

Occupational therapy specific treatment in cognitive rehabilitation often involves compensatory strategies such as schedules, reminders, cues, and environmental modifications. Additionally, occupational therapy intervention involves task accomplishment by repeated practice or simplification of functional tasks in a clinical setting [14]. Integration of domain specificity could optimize functional outcomes. For example, targeting performance patterns could improve habits (e.g., CogSMART [9]), training of performance skills helps improve the organization (e.g., GMT [1]), and consideration of contextual factors could be part of life skills training (e.g., CST [20]). Practitioners may also incorporate cognitive remediation through metacognitive strategies such as those found in GMT and SMART.

## 5. Conclusion

Researchers and clinicians across disciplines including occupational therapy practitioners, neuropsychologists, and speech pathologists are involved in addressing cognitive and functional challenges following mTBI. The OTPF helps examine the complex relationship between cognition and daily life tasks [46–48]. Therefore, integrating the OTPF in all stages of mTBI management, including characterizing and monitoring progress, could improve cognitive outcomes and optimize independent functioning.

## Figures and Tables

**Figure 1:** Articles screened and included.

**Table 1:** Database search.

	Results	Limiters
Databases		
CINAHL	188	Boolean phrase, English language, date range = 01/09-12/22, peer-reviewed, adult 19-44, middle-aged 45-64
PubMed	250	English language, publication dates = 01/09-12/22, adult 19+ years, middle-aged 45-64 years
Nursing and Allied Health	330	Keyword, English language, date range = 01/09-12/22, adult 19-44 years, middle-aged 45-64 years, peer-reviewed
Scopus	2809	Article title/abstract/keywords, date range = 2009-2022, documents, document type = all, access type = all
Trip	990	2009-2019
PsychInfo	1215	Keyword, English language, 2009-2019,
Cochrane	312	Cochrane library publication date = Jan 2009-Dec 2022, central trials only publication dates = 2009-2019, trials, word variations
Web of Science	1894	Date range = 01/01/09-12/31/22, topic search, i.e., all fields keyword
Ovid Emcare	662	Date range = 01/01/09-current, English language
Total	8650	

Electronic journals		
The Open Journal of Occupational Therapy	0	Scope of journal online in CINAHL is since 2015, date range = last four years, English language, peer-reviewed
British Journal of Occupational Therapy	32	Scope of journal online in SAGE premier is since 1999, date range = last ten years
Canadian Journal of Occupational Therapy	13	Scope of journal online in sage premier is from 1999, date range = last ten years
Occupational Therapy Now	0	Scope of journal online in nursing and allied health is from 2007, date range = last ten years, peer reviewed, English language
Australian Journal of Occupational Therapy	35	Scope of journal online in Wiley online library is since 1997, date range = last ten years, English language, peer-reviewed
Indian Journal of Occupational Therapy	0	Scope of journal online in academic search complete is since 2007, date range = last ten years, English language, peer-reviewed
Journal of Occupational Therapy Education	0	Scope of journal online in DOAJ is since 2017, date range = last three years
New Zealand Journal of Occupational Therapy	0	Scope of journal online in CINAHL is since 2003, date range = last ten years, English language, peer-reviewed
American Journal of Occupational Therapy	3	Scope of journal online in OVID is since 2000, keyword search
Scandinavian Journal of Occupational Therapy	1	Scope of journal online in CINAHL is since 1999, date range = last ten years, English language, peer-reviewed
Journal of Head Trauma Rehabilitation	57	Scope of journal online in LWW high impact collection is since 1999, date range = last ten years, English language, peer reviewed
Brain and Cognition	34	Scope of journal online in Elsevier SD freedom collection is since 1995, date range = last ten years
Total	175	

Grey literature		
Global Health: http://www.cabi.org/publishing-products/online-information-resources/global-health/	0	
Open Grey: http://www.opengrey.eu	4	
American doctoral dissertations: http://www.ebscohost.com/academic/american-doctoral-dissertations	28	
Clinicaltrials.Gov	194	
Open trials: https://explorer.opentrials.net	3	
Open access theses and dissertations (OATD) https://oatd.org/	103	
UK e-theses online service (EThOS) https://ethos.bl.uk/Home.do	0	
TWU open repository	0	
Total	332	

**Table 2:** Cognitive training programs' potential OTPF domains.

The article authors' aligned the OTPF domains with the identified programs' in the review						
Manualized programs and/or interdisciplinary programs	Occupation	Context	Performance patterns	Performance skills	Client factors	Findings
SMART (strategic memory and reasoning training): utilizes a top down strategy based approach to improve cognitive control functions of strategic attention, integrative reasoning, and innovation [15]	Education, work			Processing skills	Attention, executive functions	SMART was found to improve executive functions including reasoning, inhibition, and daily function [16].

GMT (goal management training): uses metacognitive strategies to improve patients' ability to organize and achieve goals in real-life situations [1]	Education			Task organization	Metacognition, executive functions	GMT saw improvement in self-reported cognitive executive function in daily life and improved performance on attention-demanding tasks [17].

CRT (cognitive rehabilitation therapy): enables the patient with a brain injury to return within reason to a normal life through reconstruction or compensation of the lost functions [18]					Self-awareness, attention, self-control	CRT obtained effects through the course of therapy but there was no transfer of capability to daily life [18].

CogSMART (cognitive symptom management and rehabilitation therapy): multimodal compensatory cognitive training intervention emphasizing habit learning and compensatory strategies in prospective memory, attention, learning and memory, and executive function [9]	Education (learning)		Habits		Memory, attention, executive functions Attention/working memory, verbal learning/memory, and novel problem solving	CogSMART found significant reductions in self-reported postconcussive symptoms as well as improvements in real-world prospective memory performance [9], QoL, and daily functioning [19]

CST (cognitive strategy training): aims to teach individual strategies that allow them to work around their cognitive deficits [20]	Education (psychoeducation)	Lifestyle strategies	Routine (planner)	Didactic presentations, discussions	Memory, attention, executive functions	CST showed signs of perceived usefulness of cognitive compensation strategies, reduced depression and cognitive symptom severity, and increased life satisfaction [20].

Compensatory cognitive training: group-session of interactive didactic presentations, in-class discussions, and activities that introduced participants to a variety of cognitive strategies and external aids [21]	Sleep, education (overlearning)		Time management	Organization	Memory, attention, executive functions goal-setting	This training saw fewer cognitive and memory difficulties as well as greater use of cognitive strategies. It also facilitated behavioral change and subjective/objective improvements in targeted cognitive domains [21].

GOALS (goal-oriented attentional self-regulation): a cognitive rehabilitation training program that targets executive control functions by teaching participants in applied mindfulness-based attention regulation and goal management strategies and applying them to real-life goals determined by the participant [22]		Apply skills/goals to real-life settings			Attention, memory, executive functions	GOALS had meaningful and lasting improvements in cognition, emotional regulation, and daily functioning [22].

Memory training: interventions include restorative approaches and compensatory approaches such as the use of an external memory aid (EMA) [10]	ADLs, education (of impairment), health management (meaningful activities), work, leisure				Memory, functional goals	This training saw sustained use of EMA when the intervention was linked with the client's functional and meaningful goals to get them to participate in the training [23].

Mindfulness-based stress reduction: a group-based intervention that practices mindfulness involving learning attention control and cultivating moment-to-moment awareness of thoughts, feelings, and bodily sensations [7]	Meditation, yoga				Attention, memory, perception, executive functions	This training saw an increase in selective and sustained attention, working memory, autobiographical memory, visuospatial functioning, and executive functioning [24],

Metacognitive strategy instruction: includes strategies to improve the capacity to analyze and synthesize information, direct corrective feedback for self-awareness issues, and group-based interventions for executive and problem-solving deficits [25]				Organization, planning	Memory, problem solve, dual-task operations, modeling, self-awareness, goal-directed behavior, self-regulation, self-monitoring, and reasoning	This instruction is recommended as a practice standard for improving goal-directed cognitive and emotional functioning [11].

Executive function rehabilitation: direct instruction to teach individuals to regulate their behavior by breaking complex tasks into steps while thinking strategically [26]	Cognitive orientation to occupational performance				Higher level cognitive, problem-solving, organization, higher order thinking, breaking complex tasks into steps	This rehabilitation was effective in teaching the skill but benefits did not appear to transfer over to real-life situations [26].

TAPAT (tonic and phasic alertness training): participants required to execute a speeded response via a single button press to all foil images and withhold response to the infrequent target image [27]					Executive function, attention, alertness	TAPAT saw improvements in untrained, complex, and effortful measures of executive function, suggesting that improvements in alertness can also facilitate improvements in higher-order cognitive operations [27].

Attention training: ranges from simple tasks such as using flashcards to improve basic attention skills to more complex tasks to improve complex attention and working memory using a variety of visual and verbal tasks [10]					Attention (focused, sustained, selective, alternating, and divided attention), memory	Attention training had strong evidence for treatment-specific effects of skill training for attention [26].

Functional/cognitive communication: communication rehabilitation program to provide opportunities for the person to rehearse his/her communication skills in situations appropriate to the context in which that person will live, work, study, and socialize [28]				Listening, speaking, writing, reading, conversation, and social interaction		While not a complete program, this stresses the importance of measuring outcomes that are meaningful for the person at a social participation level [28].

Return to work (RTW): cognitive interventions were focused on improving memory, postconcussive symptoms, and neuropsychological functioning [29]					Memory, attention, executive function	This program found compensatory cognitive strategies with supportive devices appear to be more effective than remedial strategies when facilitating RTW and community integration post TBI [29].

Computerized programs: designed to restore basic cognitive functions through computer-administered graded exercises [30]					Executive functions	No conclusive evidence supporting the use of computerized methods of cognitive rehabilitation following TBI was found with computer programs [26].

Virtual reality (VR): interactive stimulation that gives the user an opportunity to perform in an environment similar to a physical environment [31]	ADLs, IADLs (uses virtual environment), work, shopping			Task performance	Planning, time management, monitor performance, higher level function, self-awareness	Greater improvement found in executive function in the group that used VR, which may lead to improvement in the ability to perform IADL activities among people following TBI [31].

Artificial intelligence virtual reality based training program (AIVTS): an interactive, scenario-based program in which trainees must achieve an acceptable level before moving to the next one; otherwise, the level is repeated [32]					Cognitive functioning (in general)	AIVTS saw improvements in selective cognitive functioning but it did not transfer to real-world outcomes [32].

Psychoeducational vocational training system (PEVTS): a training manual given under the supervision of a vocational trainer by practicing routines, tutorials with specific instructional branches, simulations, and instructional games on problem-solving [32]					Problem-solving, following directions	PEVTS did not transfer into real-world outcomes [32].

CO-OP (cognitive orientation to occupational performance): metacognitive strategies, compensatory strategies, videoconference supports, and virtual reality environments for community reintegration [33]	ADLs, IADLs				Higher level cognitive (metacognitive strategies), attention (processing, divided), perception (tactile feedback)	CO-OP demonstrated that daily cognition can be improved by providing therapy in a patient's natural environment and through the use of technology to train skills needed for daily functioning [33].

Intensive cognitive communication rehabilitation (ICCR): classroom-style lectures, therapy, and technology training. Retraining of cognitive skills with academically focused application [34]	Education				Verbal expression, language and communication, memory	

BrainHQ, posit science computer training: exercises targeted at improving the speed and accuracy of neural information processing [35]					Cognitive composite scores	
